# Current Practice in Occupational Therapy for COVID-19 and Post-COVID-19 Conditions

**DOI:** 10.1155/2023/5886581

**Published:** 2023-05-19

**Authors:** C. von Zweck, D. Naidoo, P. Govender, R. Ledgerd

**Affiliations:** ^1^World Federation of Occupational Therapists, Switzerland; ^2^Discipline of Occupational Therapy, School of Health Sciences, University of KwaZulu Natal (Westville Campus), South Africa

## Abstract

The onset of the pandemic highlighted the need for a review of rehabilitation practices to ensure coordinated, effective, and efficient services for people affected by COVID-19. This paper reports on a global survey highlighting the delivery of occupational therapy services to people with COVID-19/post-COVID-19 condition (PCC) and makes recommendations to facilitate quality service delivery for this population. An online cross-sectional descriptive survey was developed and distributed to the global occupational therapy community via member organisations and communication channels of the World Federation of Occupational Therapists to collect information for this study. The survey obtained qualitative and quantitative data from respondents who were occupational therapists or occupational therapy assistants regarding (i) demographic characteristics, (ii) work experience with persons with COVID-19 and PCC, (iii) modes of working, (iv) education and training, (iv) occupational therapy intervention provided to persons with COVID-19 and PCC, and (v) the perceived quality of the occupational therapy services provided. Findings indicate that respondents provided a range of occupational therapy interventions for people affected by COVID-19/PCC aligned with evidence-based practice guidelines. While respondents identified a strong role for occupational therapy and generally rated their services as effective, issues related to the accessibility of their services impacted quality and user satisfaction. The study highlighted the need to advocate for access to occupational therapy to facilitate engagement in desired and needed occupations for COVID-19 survivors. Other recommendations emerging from the findings include the need to develop, disseminate, and use research evidence for guiding services for people with COVID-19/PCC, create quality service standards, and ensure the availability of necessary resources and supports such as referral pathways and screening criteria, availability of staff, training, personal protective equipment, and assistive devices and technology.

## 1. Introduction

COVID-19 has disrupted healthcare. This disruption highlighted the need for a review of rehabilitation practices to ensure coordinated, effective, and efficient services, which required innovation of established health delivery systems [1]. Globally, the World Health Organization (WHO) has reported *651,918,402* confirmed cases of COVID-19 [2]. In addition, many COVID-19 survivors have developed post-COVID-19 condition or PCC.

PCC occurs in individuals with a history of probable or confirmed COVID-19 infection, usually within three months from the onset of COVID-19, with symptoms that last for at least two months and cannot be explained by an alternative diagnosis. Symptoms often persist from the initial illness period ([3]: 104). People with PCC present with varied symptoms, which can occur individually or in clusters. These symptoms can be interconnected and persist for more extended periods or present as relapsing and remitting. Acknowledged symptoms affect cognition, breathing, and mental health and include fatigue, postexertional symptom exacerbation, orthostatic intolerance, and difficulties with daily living activities and returning to work [1, 3]. PCC often disrupts the ability of people to engage in their daily routine or contribute to their families and communities [4–8].

Shortly after the start of the COVID-19 pandemic in 2020, literature began to emerge regarding the benefits of rehabilitation for persons affected by COVID-19 [3, 9–11]. Acute care hospitals now often provide services for people with COVID-19 to address respiratory rehabilitation, endurance retraining, and rehabilitation for activities of daily living and instrumental activities of daily living [3]. However, there remains limited literature on the rehabilitation of persons with PCC, despite calls for integrated multidisciplinary rehabilitation at different service levels to mitigate the multisystem effect that PCC has on occupational functioning. While occupational therapists are acknowledged as part of the multidisciplinary team in the models of care for PCC in several studies [12–16], there is a paucity of literature that explores the nature of their role.

WFOT, as the global professional organisation representing 107 national occupational therapy associations across the world, embarked on research to gain insight into the provision of occupational therapy services to people with COVID-19/PCC. Additionally, WFOT sought to understand the needs of the occupational therapy community to plan for the development of future resources and support for therapists providing services to persons with COVID-19/PCC. This paper reports on a global survey that highlights the delivery of occupational therapy services to people with COVID-19 and PCC and makes recommendations to facilitate quality service delivery for this population.

## 2. Method

To collect data for this study, a cross-sectional descriptive survey was developed and hosted on SurveyMonkey®. The survey was created in English and translated by WFOT volunteers to be available in Spanish, French, and German. Each translation was reviewed by a second translator to ensure quality.

The survey was conducted between March and May 2022. A link to the online survey was distributed to the global occupational therapy community via WFOT member organisations and the WFOT website, e-news, and social media. To be eligible to complete the survey, respondents were required to be occupational therapists or occupational therapy assistants who provided occupational therapy services to people affected by COVID-19/PCC.

The 16-item survey for this study collected quantitative data via closed-ended questions using a five-point Likert scale. The questions requested information from respondents regarding (i) demographic characteristics, (ii) work experience with persons with COVID-19 and PCC, (iii) modes of working, (iv) education and training, (iv) occupational therapy intervention provided to persons with COVID-19 and PCC, and (v) the perceived quality of the occupational therapy services provided. One open-ended question asked for general comments regarding the quality of services provided to persons with COVID-19/PCC.

Responses to the survey were anonymous. The first page of the online survey provided a description of the study, and consent was obtained from all participants before starting the survey. Full approval was received for the study from the Humanities and Social Sciences Research Ethics Committee of the University of KwaZulu Natal (reference number HSSREC/00004675/2022).

Data were analysed for the study using Excel 2019 and the Statistical Package for Social Scientists version 27. The findings were stratified using variables regarding length of work experience and country income. The World Bank Classification was used to identify the income level of the countries of the respondents. The independent samples Kruskal-Wallis test was used to assess for significant differences between variables relating to working experience. An independent-sample Mann Whitney *U* test was used to determine significant differences between the variables related to country income level.

The analysis of qualitative results began with translating comments that were not submitted in English. The online Google Translate® tool was used, and any uncertainties with translations were reviewed with a native speaker. An inductive content analysis approach was adopted, letting each theme emerge through the data using inductive reasoning and constant comparison. Open codes were used to describe all the content, and codes referring to the same phenomenon were grouped into themes.

## 3. Results

### 3.1. Demographic Profile of the Respondents

A total of 740 responses were received from 69 countries. The majority of the respondents lived in high-income countries (73.1%). The survey was most frequently completed in English (48%) or German (24%), with 14% of the respondents completing the survey in Spanish or French. A large number of the respondents were practitioners (81%) or educators (15%). More than half of the respondents had 10 or more years of experience in occupational therapy (54.7%); an additional 16.4% had more than five years of experience.

### 3.2. Provision of Services for People with COVID-19 and PCC

#### 3.2.1. Training for the Provision of Services for COVID-19 and PCC

The majority of the respondents (70%) reported a sufficient amount of training for their work with people with COVID-19/PCC. Such training may have addressed specific occupational therapy interventions for this population or more generic information on topics such as infection control procedures and the pathogenesis of COVID-19. Thirteen percent of the respondents indicated that no special training was necessary. The respondents received training for their work online by webinar or e-learning (45%), peer-to-peer demonstration or supervised practice (23%), mentoring (19%), or entry-level education (16%). More than one-quarter of the respondents (28%) did not report any specific training regarding the provision of occupational therapy for people with COVID-19/PCC.

#### 3.2.2. Practice Description

Services provided by the respondents for people with COVID-19 and PCC were most often provided with public funding (48%) or with mixed public/private financing (26%). The large majority of the respondents (88%) worked with other populations in addition to sometimes or occasionally providing services to people with COVID-19/PCC. Respondents were more likely to provide occupational therapy for people with COVID-19 when compared with PCC; 75% of the respondents provided intervention as a result of a diagnosis of COVID-19, and 61% stated that individuals were seen for other issues but had COVID-19 as a comorbidity. Less frequently, respondents provided intervention as a result of a diagnosis of PCC (41%).

Services relating to COVID-19/PCC were mainly offered by the respondents in a facility such as a hospital (43%), outpatient clinic (36%), or rehabilitation centre (32%). On average, respondents indicated that 71% of them work with people with COVID-19 and PCC occurred in person. Remote intervention was less frequently provided by video conference (average 6% of working time), telephone (6%), or email/text/SMS (4%).

Average scores indicated that respondents “very often” worked with physiotherapists, doctors, and nurses in the provision of rehabilitation. “Often,” the rehabilitation team included social workers, speech-language pathologists, and occupational therapists from other settings.

Table 1 highlights the differences among team members for managing COVID-19/PCC in high- and low-/middle-income countries. Higher rates of involvement of support workers such as therapy assistants and technicians were reported in low-/middle-income countries, as well as teachers, orthotists, prosthetists, and speech therapists.

### 3.3. Occupational Therapy Interventions for People with COVID-19/PCC

When asked to describe occupational therapy services provided for individuals to address health issues specifically associated with COVID-19 or PCC, respondents reported that they provided multiple types of interventions (Figure 1). On average, respondents provided interventions “often” or “very often” in all areas assessed in the survey, except for assistive technology use, service coordination and referral, and dysphagia/swallowing disorders.

### 3.4. Quality of Service

On average, respondents rated the effectiveness of the service they provide as “high” or “very” high for the interventions they frequently provide for people with COVID-19/PCC (Figure 2). The effectiveness of occupational therapy was rated as “medium” for less frequently provided interventions including pain management, service coordination, sleep management, assistive technology use, and dysphagia management.

Access to services by occupational therapists was identified by the respondents as an area of dissatisfaction for 40% of service users. Respondents indicated that the availability of occupational therapists, wait time for occupational therapy, staff time availability, and funding of occupational therapy services were common factors that negatively impacted the quality of service (Figure 3). Although less frequently reported, important personal safety concerns were reported by 29% of the respondents, with the availability of supplies such as personal protective equipment rated with a negative impact by 24%. The identification of screening and referral mechanisms was rated most highly to positively impact the quality of service, in addition to the availability of resources such as staff time, assistive devices, and other supplies.

Comments provided by the respondents were grouped into six themes regarding occupational therapy, including poor role recognition, low funding and resources, high demand, service satisfaction and benefits, and service development/delivery. Many respondents discussed the challenges associated with the recognition of the role of occupational therapy, particularly for people with PCC, and the subsequent restrictions of funding and other resources to effectively provide services. Respondents identified a strong role for occupational therapy given the needs of people affected with COVID-19/PCC to develop self-management skills for reengaging in their daily activities. The respondents found their work rewarding, with positive feedback provided by service users, but noted that occupational therapists needed to use initiative and ingenuity to develop their services in this new area of practice. The provision of services was reported to be best suited to occupational therapists with experience and wisdom gained from working with many population groups to have the knowledge and insight needed to address the spectrum of issues and complexity of symptoms faced by people with COVID-19/PCC.

### 3.5. Association between Work Experience and Service Delivery Variables

A significant association was identified between the three service delivery variables (in-person service delivery, teleoccupational therapy service delivery, and provision of occupational therapy intervention for PCC) and the years of working experience of the respondents (Table 2). Respondents who worked <9 years chose more often to use in-person service delivery, and those with ≥10 years of work experience preferred to use teleoccupational therapy (videoconference, telephone, or email/text). Respondents who had work experience between 6 and >10 years significantly preferred to provide occupational therapy services for people with PCC.

### 3.6. Association between Country Income Class and Service Delivery Variables

There was a significant association between country income class and service delivery variables relating to the use of teleoccupational therapy services, provision of occupational therapy interventions for COVID-19 and PCC, and effectiveness of occupational therapy (Table 3). Respondents in low-/middle-income countries reported higher levels of use of teleoccupational therapy services and more frequently provided occupational therapy interventions for people with COVID-19 and PCC. The effectiveness of occupational therapy interventions was also rated more highly by respondents from low-/middle-income countries.

## 4. Discussion

This study sought to describe current global occupational therapy practice in the management of COVID-19 and PCC to make recommendations for quality service delivery. Findings indicate that respondents provided a range of interventions directed towards enhancing the ability of people affected by COVID-19/PCC to engage in desired and needed daily activities. The most common interventions provided by respondents focused on fatigue management, cognition, relaxation, self-management, environmental adaptation, and mental health. The interventions are in alignment with services recommended by the World Health Organization (WHO) in the *Clinical Management of COVID-19: Living Guideline* and the presenting symptoms documented over the last three years on the presentation of COVID-19 [1, 3, 17–20].

The interventions provided by the respondents are interrelated and overlap as depicted in Figure 4, with the outcome of each potentially affecting progress in other areas of recovery. Research evidence supports that such interventions as fatigue, breathlessness, memory and concentration problems, and pain are known to likely disrupt daily occupational functioning, resulting in a higher burden of care [3].

Brown and O'Brien [21] recommended that PCC be considered an episodic illness with multidimensional symptoms that can change unpredictably, negatively affecting the ability of people to engage in activities of daily living, community reintegration, and work. Both Brown and O'Brien [21] and WHO [3] stated that it is essential to offer a goal-oriented, person-centred approach to rehabilitation to address the impact of impairments for occupational functioning and the effect of episodic disability. Such recommendations are congruent with the basic tenets of person-centredness in occupational therapy for forming partnerships with service users to identify and implement intervention goals and strategies.

Occupational therapy services were reported in this study to be provided by a public or a public/private mix of funding, often as part of a rehabilitation team approach in a hospital, outpatient clinic, or rehabilitation centre. This finding may be a result of the larger representation of high-income respondents, where well-established public-funded healthcare systems exist. The results are aligned with the findings of Décary et al.'s [22] scoping review which highlighted the current offering of rehabilitation services for people with COVID-19/PCC across the care continuum from primary healthcare to tertiary hospitals, provided by multidisciplinary teams including physiotherapists, occupational therapists, and psychologists. The *WHO Rehabilitation Guidelines for COVID/PCC* [3] also recommends a coordinated transdisciplinary team approach that may extend to services from community healthcare workers, volunteers, and other government services such as social welfare.

Consistent with the study findings, the WHO guidelines recommend rehabilitation staff be experienced to comprehensively assess rehabilitation needs and offer support and guidance on the self-management of individual patients and their families [3]. The majority of the respondents in this survey had over five years of working experience in occupational therapy, although approximately one-third (30%) indicated that they had insufficient training for their work in this area of practice. This finding highlights the importance of research and continuing professional education supports, particularly to ensure the integration of the best available evidence in the design and provision of services for people with COVID-19/PCC. Professional organisations, employers, and individual practitioners all have a role in the development, offering, and use of such supports.

Generally, respondents perceived the occupational therapy interventions they provide as effective, with many commenting on the importance of their role and user satisfaction regarding their services. Factors negatively impacting the quality of occupational therapy centred on access to services which were limited by funding and availability of staff resources and supplies such as assistive devices and personal protective equipment. Long wait lists, high caseloads, and lack of supplies were reported in countries of all income levels, with respondents commenting that the resulting delayed and fragmented services impacted the outcomes users were able to attain. To improve access to services, the utilisation of support workers, as well as teleoccupational therapy, was reported, particularly in low-/middle-income countries. Teleoccupational therapy was used most extensively by more experienced practitioners. The availability of tools such as referral criteria and pathways was recommended to prioritise services, as well as advocacy to ensure that available services are adequately resourced. Such advocacy is necessary to build awareness of the benefits of occupational therapy and other rehabilitation services for people with COVID-19/PCC. Despite evidence-based international recommendations for the provision of rehabilitation interventions [3], respondents indicated that a low awareness existed among other health professionals regarding nonpharmacological interventions, particularly for those affected by PCC.

The authors are cognisant that the management of the long-term effects of COVID-19 was not the focus in the initial stages of the pandemic, as attention was heightened to saving lives and creating vaccines. As the pandemic progressed, however, there has been a surge in PCC conversations/discourse. Social media is flooded with accounts of how individuals cope with the long-term sequelae of COVID-19/PCC and the subsequent effect on their quality of life. With this emphasis comes the need for occupational therapists to position themselves firmly and with interventions that cover the broad spectrum of COVID-19/PCC. Hoel et al. [23] suggested the need for collaboration to promote the need for COVID-19 survivors to have access to occupational therapy and develop standards to promote quality service delivery and, in this way, reduce occupational injustice for those affected by the disease.

Results of this survey indicate that the health systems in which care is provided for people with COVID-19 have evolved significantly since the early days of the pandemic when the WFOT study was conducted by Hoel et al. [23]. During this early chaotic period, occupational therapists struggled to deliver occupational therapy services as a result of factors such as redeployment, service restrictions, and lack of preparedness with personal protective equipment, infection control procedures, and intervention guidelines and training. While rehabilitation services have developed for people with COVID-19/PCC in the intervening period, this study indicates that access and awareness of the benefits of the intervention remain a concern. We hope that the findings of this study are a catalyst for future studies that will strongly establish the role of occupational therapy in the field with the contextual nuances required for different contexts.

## 5. Limitations

Although the survey was sent to all member organisations of WFOT, a lower response rate was received compared to a previous survey sent out by WFOT on the topic of COVID-19 at the outset of the pandemic [23]. Moreover, the survey received a higher representation of high-income countries that naturally skewed the results to favour such contexts. The response may be attributable to factors such as respondent fatigue in COVID-19-related research [24], a lowered sharing of the survey with potential respondents, or a lack of required technological structure in some contexts. The lack of availability of the survey in languages other than English, French, German, and Spanish also likely restricted participation.

## 6. Conclusion

The results of this study indicate that a range of interventions are provided by occupational therapy that are aligned with the evidence-based WHO COVID-19/PCC Guidelines [3]. While respondents identified a strong role for occupational therapy and generally rated their services as effective, issues related to the accessibility of their services impacted quality and user satisfaction. The study highlighted the need to advocate for access to occupational therapy to facilitate engagement in desired and needed occupations for COVID-19 survivors. Other recommendations emerging from the findings include the need to collaborate to develop, disseminate, and use research evidence for guiding services for people with COVID-19/PCC, create standards for quality service delivery, and ensure the availability of necessary resources and support such as referral pathways and screening criteria, availability of staff, training, personal protective equipment, and assistive devices and technology.

## Figures and Tables

**Figure 1:** Occupational therapy interventions for people with COVID-19/PCC (*n* = 550).

**Figure 2:** Effectiveness of occupational therapy interventions for COVID-19 and PCC (*n* = 452).

**Figure 3:** Impact of factors on quality of occupational therapy services.

**Figure 4:** Common occupational therapy interventions for COVID-19/PCC.

**Table 1:** Multidisciplinary team members in high- and low-/middle-income countries.

Professional group (*n*)	High-income countries			Low-/middle-income countries		
	No (*n*, %)	Yes (*n*, %)	N/A (*n*)	No (*n*, %)	Yes (*n*, %)	N/A (*n*)
Doctor (*n* = 651)	45 (8.3)	431 (79.7)	65	10 (5.0)	153 (76.9)	36
Nurse (*n* = 651)	124 (22.9)	348 (64.3)	69	25 (12.6)	139 (69.8)	35
Occupational therapist (other setting) (*n* = 650)	114 (21.1)	338 (62.5)	89	37 (18.6)	122 (61.3)	40
Orthotist (*n* = 636)	336 (62.1)	66 (12.2)	139	73 (36.7)	66 (33.2)	60
Physiotherapist (*n* = 652)	54 (10)	417 (77.1)	70	9 (4.5)	156 (78.4)	34
Prosthetist (*n* = 650)	349 (64.5)	67 (12.4)	125	54 (27.1)	51 (25.6)	57
Rehabilitation/therapy assistant (*n* = 650)	242 (44.7)	168 (31.1)	131	54 (27.1)	88 (44.2)	57
Social worker (*n* = 650)	133 (24.6)	321 (59.3)	87	43 (21.6)	105 (52.8)	51
Speech therapist (*n* = 650)	171 (31.6)	290 (53.6)	58	30 (15.1)	134 (67.3)	35
Teacher (*n* = 653)	362 (66.9)	51 (9.4)	128	91 (45.7)	50 (25.1)	58
Technician (*n* = 650)	341 (63.0)	74 (13.7)	126	101(50.8)	42 (21.1)	56
Volunteer (*n* = 650)	325 (60.1)	87 (16.1)	129	99 (49.7)	39 (19.6)	61

**Table 2:** Association between work experience and service delivery variables.

	Working experience			*p* value
	<5 years Median (IQR)	6-9 years Median (IQR)	≥10 years Median (IQR)	
In-person service delivery	100.0 (60.0-100.0)	100.0 (70.0-100.0)	80.0 (30.0-100.0)	<0.001
Teleoccupational therapy service provision	0.0 (0.0-20.0)	0.0 (0.0-20.0)	10.0 (0.0-30.0)	<0.001
Specific training received to work with persons with COVID-19 and PCC	1.0 (1.0-2.0)	1.0 (1.0-2.0)	1.0 (1.0-2.0)	0.459
Provision of occupational therapy intervention for COVID-19	28.0 (18.0-35.0)	26.0 (7.3-36.0)	29.0 (13.0-37.0)	0.496
Provision of occupational therapy intervention for PCC	27.0 (19.0-36.0)	32.0 (23.8-39.0)	32.0 (23.5-38.0)	0.004
Ability to provide quality occupational therapy	25.0 (17.0-31.0)	19.0 (16.0-29.0)	22.0 (16.0-29.0)	0.123
Level of user satisfaction with service access	3.0 (2.0-3.0)	3.0 (2.0-3.0)	3.0 (2.0-4.0)	0.556
Effectiveness of occupational therapy	39.0 (28.3-49.0)	43.0 (33.0-52.0)	42.0 (32.5-51.0)	0.062

**Table 3:** Association between country income class and service delivery variables.

	Country income class		*p* value
	High-income countries Median (IQR)	Low-/middle-income countries Median (IQR)	
In-person service delivery	90.0 (40.0-100.0)	90.0 (50.0-100.0)	0.792
Teleoccupational therapy service provision	0.0 (0.0-20.0)	10.0 (0.0-40.0)	<0.001
Specific training received to work with persons with COVID-19 and PCC	1.0 (1.0-2.0)	1.0 (1.0-2.0)	0.480
Provision of occupational therapy intervention for COVID-19	25.0 (5.5-34.0)	36.0 (29.8-42.0)	<0.001
Provision of occupational therapy intervention for PCC	28.0 (20.0-35.0)	36.0 (30.5-42.0)	<0.001
Ability to provide quality occupational therapy	22.0 (16.0-29.0)	23.5 (17.0-32.0)	0.134
Level of user satisfaction with service access	3.0(2.0-3.0)	3.0 (2.0-4.0)	0.094
Effectiveness of occupational therapy	38.0 (29.0-48.0)	47.0 (39.8-54.0)	<0.001

## Data Availability

Data supporting the conclusions of this study can be accessed at https://wfot.org/resources.
